The article "The role of phagocytic leukocytes following flexible ureterenoscopy, for the treatment of kidney stones: an observational, clinical pilots-study" was published in 2020. Journal: Eur J Med Res.

# The role of phagocytic leukocytes following flexible ureterenoscopy, for the treatment of kidney stones: an observational, clinical pilots-study

**DOI:** 10.1186/s40001-020-00466-7

**Published:** 2020-12-11

**Authors:** Stephen Fôn Hughes, Alyson Jayne Moyes, Rebecca May Lamb, Peter Ella-tongwiis, Nana Yaa Frempomaa Snyper, Iqbal Shergill

**Affiliations:** 1 North Wales and North West Urological Research Centre, Betsi Cadwaladr University Health Board (BCUHB) Wrexham Maelor Hospital, Wrexham, Wales UK; 2 North Wales Clinical Research Centre, Betsi Cadwaladr University Health Board (BCUHB) Wrexham Maelor Hospital, Wrexham, Wales UK; 3 School of Medical Sciences, Bangor University, Bangor, Wales UK; 4 Department of Urology, BCUHB Wrexham Maelor Hospital, Wrexham, Wales UK

**Keywords:** Flexible ureterenoscopy, (FURS), Flow cytometry, Kidney stones, Inflammation, Biomarkers, Leukocytes

## Abstract

**Background:**

The number of patients undergoing flexible ureterenoscopy (FURS) for the treatment of kidney stones (renal calculi) is increasing annually, and as such the development of post-operative complications, such as acute kidney injury (AKI), haematuria and infection is likely to increase. Phagocytic leukocytes are white blood cells that help fight foreign material such as bacteria and viruses, and they are intrinsically involved in the inflammatory reaction. Investigating the role of phagocytic leukocytes following FURS has not been widely researched. The main aim of the study was to evaluate the role phagocytic leukocytes (neutrophils and monocytes) function, in patients undergoing FURS for the treatment of kidney stones (renal calculi).

**Methods:**

Fourteen consecutive patients aged between 27 and 70 years (median 49.5 years) undergoing FURS for the treatment of kidney stones were recruited (seven males, seven females). Blood samples were collected from each patient at four time points: baseline (pre-operatively) followed by 30, 120 and 240 min post-operatively. Mononuclear (MN) and polymorphonuclear (PMN) leukocyte sub-populations were isolated by density gradient centrifugation techniques. Neutrophil and monocyte cell function was investigated by measuring the cell surface expression of CD62L (L-selectin), CD11b (Mac-1), CD99 and the intracellular production of hydrogen peroxide (H_2_O_2_), via flow cytometry.

**Results:**

Significant increases was observed in monocyte CD62L expression post FURS for the treatment of kidney stones (*p* ≤ 0.05); while significant decreases were observed in neutrophil CD62L. The levels of the other activation markers CD11b, CD99 and H_2_O_2_ corresponded to the increases and decreases seen in CD62L for monocytes and neutrophils respectively, though the changes were not statistically significant (*p* > 0.05). Limiting factors for this study were the relatively small sample size, and restriction on the recruitment time points.

**Conclusions:**

This study demonstrates that following FURS for the treatment of kidney stones, monocytes are rapidly activated and produce potent reactive oxygen intermediates. Interestingly, the pattern of expression in neutrophils suggests that these cells are deactivated in response to the treatment. The leukocyte biomarkers assessed during this investigation may have a role in monitoring the ‘normal’ post-operative response, as no complications occurred in any of the patients; or may help predict potential infectious complications (e.g. urosepsis) that can occur during the post-operative period. This data, however, will need to be validated and reproduced in larger multi-centre studies.

## Background

Kidney stone disease (nephrolithiasis) contributes to a significant proportion of routine urological practice and remains a common cause of worldwide morbidity [1]. Globally, the average lifetime risk of developing kidney stones (renal calculi) is 5–10% [2]. However, industrialised countries exhibit higher incidence rates, with the male lifetime risk of developing kidney stones being 18.8% and the female risk being 9.4% [3]. Alarmingly, both the incidence and prevalence of kidney stones continues to rise, irrespective of age, race or gender [4–7]. Furthermore, it can be appreciated that with an increase in kidney stone incidences, comes an increase in the demand for treatment, which in turn, escalates the proportion of patients who may develop a post-operative complication as a result of intervention.

The number of patients undergoing flexible ureterenoscopy (FURS) for the treatment of kidney stones is increasing annually. The overall complication rate after FURS is 9–25% [8]. Following FURS, there is a risk of developing post-operative complications such as infection, bleeding, renal injury, sepsis and pain [9]. With an annual increase in the number of patients undergoing FURS surgery, it is expected that the instances of such complications will also increase, and if left untreated, these complications may be fatal [10]. Although it recognised that FURS is a generally successful, minimally invasive means of removing stones, the primary consideration in managing stones must be diverted from analysing stone free rates: to instead focus on the process of removing stones with minimal complications, to reduce the incidences of associated morbidities. It is, therefore, imperative that healthcare providers have a means to confidently predict those patients who undergo surgery, who are likely to develop post-operative complications such as obstructed kidneys, infection or subsequent urosepsis.

Conventionally in the UK, patients undergoing urological surgery have been post-operatively monitored using C reactive protein (CRP) and erythrocyte sedimentation rate (ESR), which are established markers of inflammation [11]. However, the disadvantage to measuring these markers is their non-specific nature [12], resulting in an inability to differentiate between inflammations due to inter-current or pre-existing disease processes, to those arising as a direct complication of treatment or surgery.

Phagocytic leukocytes are components of the non-specific immune system. Monocytes and neutrophils are examples of phagocytic leukocytes and it can be appreciated that they play a key role during inflammation due to their adhesion, trans-endothelial migration and subsequent activation into the surrounding tissues [13, 14]. They are important cells that are able to mediate tissue damage with vital involvement in modulation of host defence via the innate immune response, they can internalise and destroy potentially harmful pathogens and infectious agents via phagocytosis [14]. Leukocytes are intrinsically involved with the vascular endothelium, and express specific adhesion molecules (e.g. CD62L, CD11b, CD99) on their cell surfaces for facilitating such interactions. During cellular activation, leukocytes produce and release potent proteolytic enzymes and reactive oxygen intermediates [13–15], which may contribute toward some of the post-operative complications that can develop following FURS. Both neutrophils and monocytes have been implicated to play a key role during the inflammatory response post-surgery and thus deserve research attention [16–18].

CD62L (L-selectin) is an adhesion molecule that is part of the selectin family. It is a cell surface glycoprotein that is expressed on the cell surface of most leukocytes. CD62L has a vital role in leukocyte migration. CD62L has a shedding mechanism, in an attempt to regulate the rate at which leukocyte extravasation occurs in inflamed tissues [19].

CD11b (Mac-1) is a member of the integrin family and is expressed on the cell surface of the majority of leukocytes, including macrophages, monocytes and neutrophils as well as natural killer cells [20]. CD11b’s functional role involves adhesion and migration of activated leukocytes in response to inflammatory stimulus [13, 21, 22].

CD99 is a glycoprotein that is expressed on most leukocyte cells. CD99 has a unique role and is involved in the homophylic interactions during trans-endothelial migration. Raised levels of neutrophil CD99 levels were recently reported in a cohort of patients with inflammatory bowel disease, thus indicating that CD99 is directly involved to inflammatory responses [23].

Hydrogen peroxide is a strong oxidising agent and is produced by phagocytic cells such as monocytes and neutrophils. Increased intracellular production of H_2_O_2_ levels has been reported following various orthopaedic surgical interventions, but as yet have not been reported following FURS [16, 17]. The present study was designed to ascertain whether FURS for the treatment of kidney stones results in changes to neutrophils and monocytes cell surface expression of the CD62L, CD11b and CD99 adhesion molecules, and to assess the intracellular production of H_2_O_2_.

Whilst we, and others, have previously reported post-operative changes in routine blood tests (haematological and biochemical) following various urological surgical procedures [24–26], crucially, there is very little evidence investigating the direct effect of FURS on leukocyte function. An important aspect of this clinical pilot-study was to provide a better understanding of the role of phagocytic leukocytes following FURS. Specifically, we aimed to evaluate changes in leukocyte function to provide a better understanding of their post-operative course following elective FURS, for the treatment kidney stones. It was our expectation to enhance current urological literature by adding a evidence based insight on this topic, and to provide findings that may ultimately aid clinicians in distinguishing the ‘normal’ post-operative response to those at increased risk of complications such as infection following FURS; however, the validation and reliability needs to be assessed through larger cohort studies.

### Methods

#### Subject volunteers

Ethical approval for this study was received from the Welsh Research Ethics Service (REC) 4 committee (REC4: 12/WA/0117). Fourteen consecutive patients, scheduled for elective FURS for the treatment of kidney stones were recruited (*n* = 14). Specifically, seven males and seven females aged between 27 and 70 years (median 49.5 years) were recruited after receiving written informed consent.

#### Flexible ureterenoscopy (FURS) and blood collection

Treatment was given as per standardised protocol at the Betsi Cadwaladr University Health Board (BCUHB) Wrexham Maelor, NHS hospital, North Wales, UK under the same consultant urologist. An Olympus P5 Flexible Ureterorenoscopy was used during the surgery, while patients were under general anaesthesia using Propofol. The mean FURS procedure time was 58 min (22–104 min). Complete stone clearance was achieved in all patients, with no complications reported post-treatment.

Prior to FURS, a venous blood sample was collected pre-operatively from the arm via the antecubital fossa Blood samples were collected into di-potassium ethylene diamine tetra-acetic acid (EDTA), which stood as a baseline (control) measurement. The baseline (pre-operative) samples served as the control measures during this study, with the main aim being to compare the effects of FURS on the leukocyte parameters measured within each subject pre and post-operatively.

Following FURS, further blood samples were taken at 30, 120 and 240 min post-operatively. The fresh blood samples were then isolated within 4 h and used for flow cytometric analysis of Cluster of Differentiation (CD) markers: CD99, CD11b, CD62L and intracellular production of H_2_0_2_.

With regards to the choice of anticoagulant used during blood collection procedures in the present study, previous studies have reported that blood collected in heparin lead to cellular activation and increased expression of CD11b in comparison to cells in blood drawn into EDTA [27]. Interestingly, Patil et al. [28] found that the levels of a number of cytokines (i.e. IL-6, IL-8, IL-10, IL-17, MIP-1β, GM-CSF and MCP-1) were significantly higher in blood samples collected in heparin compared to those collected in EDTA. With regard to the present study, all blood samples were collected into EDTA vacutainers to avoid any unnecessary leukocyte activation.

#### Isolation of leukocytes

Phagocytic leukocytes were isolated from whole blood samples. The blood was collected in EDTA vacutainers, and the mononuclear cell (MN) and polymorphonuclear cells (PMN) were separated using a density-gradient centrifugation method using Ficoll-Hypaque solutions supplied by Sigma, UK.

Isolated PMN and MN were then counted using a Beckman Coulter DxH 500 (Beckman Coulter, UK) to establish the purity and total numbers (Fig. 1). Subsequently, cell counts were adjusted to 2 × 10^6^ cells/ml with PBS/EDTA before immediate measurement using the Becton Dickinson (BD) Accuri C6 flow cytometer (Beckman Dickinson, New Jersey, USA), which had been initially validated and gated for the analysis of leukocyte subpopulations (Fig. 2). The isolated cells were analysed within 4 h to ensure live cell viability.

**Fig. 1:** Efficiency of leukocyte isolation methods. Percentage yields of MN and mononuclearand PMN granulocyte cells was calculated following measurement using a Beckman DxH 500. Results are presented as means ± SD

**Fig. 2:** Example gating of leukocyte subpopulations during flow cytometric analysis, employing the BD Accuri C6 flow cytometer

#### Measurement of cell surface expression of CD62L, CD11b and CD99

Commercially optimised monoclonal antibodies used were mouse anti-human CD99 (MCA1850), CD62L (MCA1076F) and CD11b (MCA551F), along with their isotype-matched controls. All reagents were purified immunoglobulin/fluorescein isothiocyanate (Ig/FITC) conjugates supplied from Bio-Rad, UK (formerly AbD Serotec).

Isolated leukocyte subpopulations PMN and MN were incubated in monoclonal antibodies at 0.1 mg/ml for 30 min at room temperature, prior to assay analysis using flow cytometry of gated monocytes and neutrophils (Fig. 2). Changes in the cell surface expression of CD62L, CD11b and CD99 (represented by mean fluorescent intensity) were measured at each time interval to assess the effect of FURS on phagocytic cell function.

#### Measurement of intracellular hydrogen peroxide production (H_2_O_2_)

Cells were isolated and intracellular H_2_O_2_ production was assessed by adaptation of a technique originally described by Bass et al. [30]. The assay was based on the oxidation of non-fluorescent 2′, 7′-dichlorofluoroscin diacetate (DCFH-DA) by H_2_O_2_ to stable and fluorescent dichlorofluoroescein. H_2_O_2_ production was assessed in cells using a fixed volume of 0.5 ml cell suspension (2 × 10^6^ cells/ml) mixed with 0.5 ml DCFH-DA (20 µM) in PBS. Cells were incubated in the dark, at 37 °C for 30 min before immediate measurement using flow cytometry of gated monocytes and neutrophils (Fig. 2).

#### Statistical analysis

Statistical analysis for this clinical pilot-study was carried out using SPSS for Windows, version 24. Initial testing for normal distribution was carried out on all sample populations, with results being measured against the Kolmogorov–Smirnov, with data being classified as normally distributed if *p* ≥ 0.05*.*

Where data were parametric, repeated measures one-way analysis of variance (ANOVA) between samples test was employed, adopting a 5% level of significance. Post hoc testing was conducted using the Bonferroni test for pairwise comparisons between means. All parametric data are presented as mean ± standard deviation (SD).

Data that did not comply with normality were analysed using the Friedman test. Where the Friedman test resulted in statistical significance, subsequent tests were performed using the Wilcoxon test. Statistical significance was accepted when *p* ≤ 0.05. All non-parametric results are presented as median ± interquartile range (Iqr).

## Results

### Efficiency of the leukocyte isolation method

The efficiency of the leukocyte isolation method is illustrated in Fig. 1***.*** The percentage isolation yield of the mononuclear (monocyte and lymphocyte) cells (94.2 ± 12.7%) was slightly higher than that for the PMN cells (90.9 ± 6.73%). The low erythrocyte presence in the isolated cells (0.01 ± 0.002%) indicates that the isolation method was effective, as there is minimal contamination of red blood cells present. The isolated MN and PMN cell populations were subsequently analysed via flow cytometry.

### The effect of FURS on CD62L cell surface expression of neutrophils and monocyte

The results are expressed as Mean Fluorescent Intensity (MFI) and represent changes to the CD62L cellular surface expression in both neutrophils and monocytes, both pre-operatively (baseline) and after FURS (30, 120 and 240 min post-operatively), for the treatment of kidney stones.

ANOVA analysis results show a statistically significant decrease in the expression of CD62L in neutrophils, *p* = 0.042 (Fig. 3). Baseline levels of CD62L, (38,554 ± 2,644 MFI), increased at 30 (45,715 ± 4,661 MFI), then decreased at 120 (42,130 ± 2,902 MFI) and 240 min post-op (36,610 ± 2,988 MFI). Post hoc Bonferroni testing showed that there was no significant difference in the production of H_2_0_2_ between baseline vs 30, 120 and 240 min post-FURS (*p* > 0.05).

**Fig. 3:** Effect of flexible ureterenoscopy on CD62L cell surface expression of neutrophils and monocytes. The points represent mean ± SD

The CD62L cell surface expression on monocytes increased from the baseline value (40,828 ± 32,29 MFI) following FURS at 30 (53,107 ± 4299 MFI), 120 (60,732 ± 7,643 MFI), and decreased at 240 min post-op (58,402 ± 7,861 MFI). The increasing pattern observed in CD62L cell surface expression on monocytes, was found to be significant using ANOVA testing *p* = 0.006 (Fig. 3). Post hoc Bonferroni testing showed that there was significant difference in CD62L between baseline vs 30 (*p* = 0.023), 120 (*p* = 0.011) and 240 (*p* = 0.08) minutes post-FURS.

### The effect of FURS on CD11b cell surface expression of neutrophils and monocytes

The results are expressed as Mean Fluorescent Intensity (MFI) and represent changes to the CD11b cellular surface expression in both monocytes and neutrophils, both pre-operatively (baseline) and after FURS (30, 120 and 240 min post-operatively), for the treatment of kidney stones.

Friedman analysis results showed no statistically significant increases in the expression of CD11b in neutrophils, *p* = 0.593 (Fig. 4). Baseline levels of CD11b (45,547 ± 36,839 MFI), decreased at 30 (36,300 ± 31,090 MFI), and increased at 120 min (40,240 ± 31,432 MFI) and at 240 min post-operatively (40,978 ± 24,717 MFI).

**Fig. 4:** Effect of flexible ureterenoscopy on CD11b cell surface expression of neutrophils and monocytes. The points represent median ± Iqr (neutrophils) and mean ± SD (monocytes)

The CD11b cell surface expression on monocytes increased from the baseline (51,873 ± , 5,031 MFI) following FURS at 30 (57,691 ± 6,316 MFI) and at 120 (60,972 ± 9,034 MFI) minutes post-operatively. At 240 min post-operatively (54,003 ± 6,638 MFI) CD11b cell surface expression decreased toward balsa levels. However, changes in CD11b cell surface expression on monocytes, was found not to be significant via ANOVA analysis *p* = 0.356 (Fig. 4).

### The effect of FURS on CD99 cell surface expression *of neutrophils and monocytes*

The results are expressed as Mean Fluorescent Intensity (MFI) and represent changes to the CD99 cellular surface expression in both monocytes and neutrophils, both pre-operatively (baseline) and after FURS (30, 120 and 240 min post-operatively), for the treatment of kidney stones.

Friedman analysis results showed no significant decrease in the expression of CD99 in neutrophils, *p* = 0.138 (Fig. 5). Baseline levels of CD99 (32,223 ± 22,728 MFI) decreased at 30 (26,830 ± 14,255 MFI), 120 (19,591 ± 16,671 MFI) and 240 min post-operatively (18,739 ± 12,934 MFI).

**Fig. 5:** Effect of flexible ureterenoscopy on CD99 cell surface expression of neutrophils and monocytes. The points represent median ± Iqr

The CD99 cell surface expression on monocytes increased initially from the baseline value (62,273 ± 57,396 MFI) following FURS at 30 min (70,173 ± 57,745 MFI), and at 120 min (81,935 ± 72,138) post-operatively. However, CD99 expression decreased at 240 min post-op (78,801 ± 67,939 MFI). However, the changes observed in CD99 cell surface expression on monocytes, were found not to be significant using Friedman testing *p* = 0.078 (Fig. 5).

### The effect of FURS on intracellular production of H_2_0_2_ of neutrophils and monocytes

The results are expressed as Mean Fluorescent Intensity (MFI) and represent changes seen in levels of intracellular H_2_0_2_ production in both monocytes and neutrophils, both pre-operatively (baseline) and after FURS (30, 120- and 240-min post-op), for the treatment of kidney stones.

Friedman analysis results showed no significant changes in H_2_0_2_ production in neutrophils, *p* = 0.082 (Fig. 6). Specifically, there was an increase from baseline levels of H_2_0_2_ (89,527 ± 54,958 MFI) at 30 min post-operatively (98,804 ± 75,880 MFI). However, there was a decrease in H_2_0_2_ production at 120 (93,227 ± 62,919 MFI) and 240 min (76,283 ± 45,955 MFI) post-operatively.

**Fig. 6:** Effect of flexible ureterenoscopy on H_2_0_2_ on cell surface expression of neutrophils and monocytes. The points represent mean ± SD (neutrophils) and median ± Iqr (monocytes)

There was an increase in intracellular H_2_0_2_ production of monocyte cells from baseline (128,102 ± 52,593 MFI) to 30 (149,953 ± 71,204 MFI) and 120 min (168,859 ± 88,390 MFI) post-operatively. However, at 240 min the H_2_0_2_ levels decreased back towards the basal value (150,951 ± 82,084 MFI). However, analysis of the data via ANOVA found the changes observed not to be significant, *p* = 0.075 (Fig. 6).

## Discussion

The main aim of this study was to evaluate the role of phagocytic leukocytes (neutrophils and monocytes) in patients undergoing FURS for the treatment of kidney stones. It can generally be appreciated that damage occurs to the vascular endothelium following FURS, due to the passage, and consequential stone removal with a flexible ureterenoscope. Consequently, it is speculated that leukocyte margination will occur at sites of trauma, subsequently leading to leukocyte activation. In order to establish the role of monocytes and neutrophils following FURS, cell surface adhesion molecules CD62L, CD11b, CD99 and intracellular production of H_2_O_2_ were assessed.

The present study reports of changes to neutrophils and monocytes cell surface expression of CD62L, CD11b and CD99 following FURS, which is associated with leukocyte cell activation (Table 1). This was further supported by the increase in intracellular H_2_O_2_ production of neutrophils and monocytes. It can also be appreciated that during leukocyte activation further bioactive material, such as other reactive oxygen intermediates (e.g. myeloperoxidase and superoxide) and proteolytic enzymes (e.g. elastase) are released extracellularly [13, 22]. Collectively, the actions of these degradative substances may potentially cause considerable damage to host tissue, prolong the inflammatory response following FURS and may play an integral role in the development of post-operative complications.

**Table 1:** Summary of main findings

Statistically significant increases were observed in monocyte CD62L expression post FURS for the treatment of kidney stones (*p* ≤ 0.05)
Statistically significant decreases were observed in neutrophil CD62L expression post FURS for the treatment of kidney stones (*p* ≤ 0.05)
No statistically significant changes were seen in neutrophils and monocytes CD11b, CD99 and H_2_0_2_ levels, post FURS for the treatment of kidney stones (*p* ≥ 0.05). Though trend mirrored CD62L
Monocytes consistently expressed more cell surface expression of CD62L, CD11b, CD99 and produced more intracellular H_2_0_2_ following FURS compared to neutrophils

With regard to the work undertaken by Moyes et al*.* [24], who evaluated changes to haematological and biochemical blood tests after FURS for the treatment of kidney stones, the present study compliments this work and provides a further insight into the role of phagocytic leukocytes pertaining to the ‘normal’ post-operative response following FURS, as no complications were reported in any of the patients in the present study. Data reported from the present study also follow a similar trend of leukocyte activation that has been previously reported by Hughes et al*.* [16, 17] following upper and lower limb orthopaedic surgeries.

We report that selective phagocytic leukocyte biomarkers such as CD62L, CD11b, CD99 and H_2_O_2_ may provide alternative ways of monitoring patients during the post-operative period following FURS. It is, therefore, proposed that by allowing urological surgeons access to these laboratory markers, an accurate assessment of the extent of inflammation following surgery per se may be made. The leukocyte biomarkers assessed during this investigation may have a role in monitoring ‘normal’ response and to help predict potential infectious complications (e.g. urosepsis) that can occur during the post-operative period.

This is the first study to report on the role of phagocytic leukocytes to following FURS for the treatment of kidney stones. However, in order to fully understand the role of phagocytic leukocytes following FURS, further studies involving larger cohorts and longer post-operative monitoring and blood sampling (e.g. 4–24 + hours) is needed. Furthermore, it is acknowledged that a limiting factor of this pilot-study is the relatively small number of participants recruited (*n* = 14). For future studies involving flow cytometry, it would be beneficial to employ monoclonal antibodies specific for a particular cell type (e.g. CD14 and CD64 for the identification of mature monocyte populations). Nevertheless, we feel that these observational findings provide encouragement for further exploration into the role of phagocytic leukocytes and its correlation with clinical outcome measures (e.g. infection), in larger cohorts following FURS. Although none of the patients during this study had an untoward outcome, it would be beneficial for future investigations to include a control other than the patients themselves, for example by comparing patients undergoing shock wave lithotripsy, which is a non-invasive procedure for the treatment of small kidney stones. This would provide an alternative control measure and help generate unique results to establish the extent of inflammation and changes to phagocytic leukocyte function following both procedures. In turn, this may also help fully understand the attributing effects that anaesthesia may have on patients’ blood for those undergoing FURS.

Ultimately, if changes to leukocyte function following FURS can identify or predict those patients at increased risk of complications such as bleeding and infection, future directions of this study may offer the potential of pharmacological intervention. For example, using anti-haemorrhagic agents as preventative measures for post-operative bleeding or providing antimicrobial agents for infection could improve patients’ recovery following FURS for the treatment of kidney stones.

## Conclusion

This study demonstrates that following FURS for the treatment of kidney stones, monocytes are rapidly activated and produce potent reactive oxygen intermediates. Interestingly, within the time points studied, it appears that neutrophils undergo down-regulation of the activation markers suggesting that their role in the response to the treatment is different from that of the monocytes. The leukocyte biomarkers assessed during this investigation may have a role in monitoring the ‘normal’ post-operative response, as no complications occurred in any of the patients; or may help predict potential infectious complications (e.g. urosepsis) that can occur during the post-operative period. These data, however, will need to be validated and reproduced in larger multi-centre studies.

## Data Availability

All data generated or analysed during this study are included in the published article.

## Abbreviations

CD marker: Cluster of differentiation marker
CD11b: Cluster of differentiation 11b (alternative name: Mac-1)
CD62L: Cluster of differentiation 62L (alternative name: L-selectin)
CD99: Cluster of differentiation 99
CRP: C reactive protein
EDTA: Ethylene diaminetetraacetic acid
ESR: Erythrocyte sedimentation rate
FITC: Fluorescein isothiocyanate
FURS: Flexible ureterenoscopy
H_2_0_2_: Hydrogen peroxide
Ig: Immunoglobulin
Iqr: Interquartile range
MN: Mononuclear cells
PMN: Polymorphonuclear cells
SD: Standard deviation
SWL: Shock wave lithotripsy
